# Nifedipine plus Systematic Nursing on Pregnancy Outcomes in Patients with Gestational Hypertension

This article has been retracted.

**DOI:** 10.1155/2022/4417790

**Published:** 2022-06-08

**Authors:** Yan Ma, Yingping Zhang

**Affiliations:** Maternity Ward of Jiangsu Hai'an County People's Hospital, No. 17 Zhongba Middle Road, Hai'an City 226600, Jiangsu Province, China

## Abstract

**Objective:**

To study the effect of nifedipine combined with systematic nursing on pregnancy outcomes in patients with gestational hypertension.

**Methods:**

According to the random number table method, 120 patients with gestational hypertension treated in our hospital were divided into the control group (60 cases) and observation group (60 cases). The control group was given magnesium sulfate treatment, the observation group was given magnesium sulfate combined with nifedipine, and the two groups of patients were given systematic nursing. The blood pressure levels, negative emotions, and pregnancy outcomes of the two groups of patients before and after treatment were compared. The blood pressure levels of the two groups before and after treatment were measured by the electronic sphygmomanometer, and the self-rating depression scale (SDS) and self-rating scale (SAS) were used to evaluate the depression and anxiety of the two groups, respectively.

**Results:**

After treatment, the systolic blood pressure, diastolic blood pressure, SDS score, and SAS score of the two groups were decreased, and the observation group was significantly lower than the control group. Additionally, the observation group had lower incidence of cesarean section, postpartum hemorrhage, premature rupture of membranes, and neonatal asphyxia (*P* < 0.05).

**Conclusion:**

Nifedipine plus systematic nursing in patients with gestational hypertension can effectively improve the pregnancy outcome and adverse emotions such as depression and anxiety, reduce blood pressure, and promote disease recovery.

## 1. Introduction

Pregnancy-induced hypertension (PIH) is a condition of increased blood pressure in pregnant women after 20 weeks of pregnancy, with early clinical manifestations of anemia, dizziness, proteinuria, increased blood pressure, and coma and convulsions in severe cases [1]. Recent years witness a rising incidence of gestational hypertension, imposing a serious threat to the safety of pregnant women and fetuses [2]. Despite the wide availability of magnesium sulfate in the treatment of gestational hypertension, its therapeutic concentration is associated with toxicity; therefore, the dosage is clinical concern and restricts its use [3]. Nifedipine is a calcium channel blocker that can relax smooth muscle, dilate blood vessels, and lower blood pressure and is often used in the treatment of hypertensive patients [4]. In clinical treatment, proper nursing measures is more conducive to the recovery of the patient's disease. Systematic nursing, with modern nursing concept as the guidance, nursing procedures as the core, involves clinical nursing and nursing management in a systematic way. It embodies the system, integrity, decision-making, and scientific nature of nursing work. Also, the systematic nursing method can intervene in the patient's diet, psychology, health education, and other aspects, which can effectively improve the patient's negative emotions [5]. From the perspective of traditional Chinese medicine, PIH belongs to the category of “blood stasis,” and its main occurrence is related to astringency stagnation, deficiency of qi and blood, and blocked blood circulation, so the treatment mainly focuses on promoting blood circulation to remove stasis, regulating channels and collaterals, calming the mind, and nourishing the body. Systematic nursing based on traditional Chinese medicine is also effective in PIH. In this study, nifedipine combined with systematic nursing was applied to treat patients with gestational hypertension.

## 2. Materials and Methods

### 2.1. Patients

According to the random number table method, 120 patients with gestational hypertension who were admitted to our hospital between June 2020 and June 2021 were assigned at a ratio of 1 : 1 either to the control group or observation group. The age of the control group was 23–45 years old, with an average of (28.85 ± 4.36) years old; the gestational age was 22–35 weeks, with an average of (28.02 ± 4.58) weeks; the disease severity: 18 cases of mild, 35 cases of moderate, and 7 cases of severe; and pregnancy history: 35 primipara and 25 multiparous. The age of the observation group was 24–47 years old, with an average of (29.85 ± 5.37) years old; the gestational age was 23–37 weeks, with an average of (29.13 ± 5.42) weeks; the disease severity: 15 cases of mild, 30 cases of moderate, and 15 cases of severe; pregnancy history: 37 primipara and 23 multiparous. The baseline data such as age, gestational age, and pregnancy history were similar in the two groups. This study has been reviewed and approved by the Medical Ethics Committee of the Jiangsu Hai'an County People's Hospital, No. HA29003. Diagnostic criteria referred to diagnosis and treatment of hypertensive diseases during pregnancy [6]. Patients were assessed as eligible if they met the above diagnostic criteria, aged between 20 and 50 years old, were conscious and willing to cooperate with the treatment, and blood pressure was above 140/90 mmHg; whereas, patients with severely abnormal heart, liver, and kidney functions, malignant tumors, with allergies to therapeutic drugs or allergic constitution, with autoimmune diseases or infectious diseases, recent use of hormones and immune preparations, with severe mental disorders, and with coagulation disorders or other blood system diseases were excluded from the study.

### 2.2. Methods

#### 2.2.1. Treatment Method

Control group: magnesium sulfate injection (Shanghai Xudong Haipu Pharmaceutical Co., Ltd., H31020666, specification: 10 mL: 2.5 g) 5 g was diluted with 20 mL of 10% glucose and injected intravenously. In addition, magnesium sulfate injection was dissolved into 500 mL of 5% glucose injection, and the drip rate was adjusted according to the patient's blood pressure, 1–1.5 g/h. Observation group: on the basis of the control group, oral nifedipine sustained-release tablets (Dezhou Deyao Pharmaceutical Co., Ltd., H10920005, specification: 10 mg/tablet) were given, 10 mg/time, 3 times/d. Both groups of patients were treated for consecutive 10 days.

#### 2.2.2. Nursing Methods

Both groups of patients were given systematic nursing on the basis of treatment. The specific methods are as follows. Health education: all patients were carefully explained by their corresponding responsible nurses on the causes of gestational hypertension, clinical manifestations, and factors affecting the occurrence of the disease and later treatment methods when they were admitted to the hospital, so that the patients could understand the relevant hazards of the disease and how to prevent the importance of improving patients' awareness of the disease and compliance with later treatment. Psychological care: a clean and comfortable ward environment should be provided, so that patients can maintain a relaxed and happy mood during hospitalization and reduce negative emotions; a good doctor-nurse relationship with patients should be established, such as listening carefully to patients' demands and needs and conducting effective communication, sending positive and optimistic emotions to patients, encouraging patients to have the confidence to overcome the disease, and reducing anxiety, depression, and other negative emotions. In addition, family members of patients should be instructed to pay more attention to accompanying patients, strengthen daily communication and exchanges with patients, and enhance patients' self-confidence. Diet care: the patient's daily diet should be intervened, such as ensuring the normal intake of high protein and vitamins every day and timely supplementing trace elements such as calcium, iron, and iodine. Vital signs monitoring: after admission, all patients should be regularly checked for urine routine, urine protein, and other indicators, and the patient's vital signs and placenta should be regularly monitored. Perinatal care: before delivery, pregnant women's blood pressure, pulse, heart rate, respiration and oxygen saturation, and other vital signs should be closely monitored, and their contractions, fetal heart rate, and vaginal bleeding should be observed. For unstable fetal heart rate or vaginal bleeding, early measures should be taken.

### 2.3. Observation Indicators

#### 2.3.1. Blood Pressure

The blood pressure of patients before and after treatment was measured by the electronic sphygmomanometer. Mindray IMEC8 color ultrasound Doppler ultrasound (purchased from Shenzhen Mindray Biomedical Electronics Co., Ltd.) was used to measure the changes of systolic blood pressure, diastolic blood pressure, and heart rate.

#### 2.3.2. Negative Emotions

The self-rating depression scale (SDS) [7] was used to evaluate the severity of depression in patients. A score of 53–62 indicates mild depression, 63–72 indicates moderate depression, and 73–100 indicates severe depression. The self-rating scale (SAS) [8] was used to evaluate the severity of anxiety. A score of 50–59 points indicates mild anxiety, 60–69 points indicates moderate anxiety, and 70–100 points indicates severe anxiety.

#### 2.3.3. Pregnancy Outcomes

The pregnancy outcomes were recorded, including cesarean section, postpartum hemorrhage, premature rupture of membranes, and neonatal asphyxia.

#### 2.3.4. Nursing Satisfaction

The self-made nursing satisfaction questionnaire was used to conduct the survey, including 5 aspects of overall service, comfortable operation environment, health education, convenient procedure, and psychological nursing, and grouped into satisfactory, modest, and unsatisfactory. Before discharge from the hospital, the specially trained nursing staff issued questionnaires, guided them to fill in the questionnaires, and collected them on the spot.

The 24-hour urine protein quantification, random urine protein/creatinine value, serum homocysteine (Hcy), and C-reactive protein (CRP) were compared between the two groups before and after treatment. After admission, 3 mL of fasting venous blood was drawn from all patients before and after treatment at 8 : 00 a.m., placed in a nonanticoagulant test tube and coagulated, centrifuged for 10 min to extract the supernatant, and then stored at −20°C for testing. The serum Hcy and CRP levels were detected by the ELISA method, and the kits were purchased from Shanghai Keen Technology Co., Ltd.

### 2.4. Statistical Methods

The SPSS 21.0 software was used for data analysis, measurement data and enumeration data are expressed as (*x* ± *s*) and *n* (%), respectively, and *t* and *χ*^2^ tests were used for comparison between groups, respectively. *P* < 0.05 was considered statistically significant.

## 3. Results

### 3.1. Comparison of Blood Pressure Levels

The data showed that the systolic blood pressure and diastolic blood pressure levels of the two groups of patients were decreased after treatment, with lower results in the observation group (*P* < 0.05), as given in Table 1.

### 3.2. Comparison of Negative Emotion Scores

The decrease of SDS and SAS scores of the patients in the two groups were significant, with lower results in the observation group (*P* < 0.05), as given in Table 2.

### 3.3. Comparison of Pregnancy Outcomes

The incidence of cesarean section, postpartum hemorrhage, premature rupture of membranes, and neonatal asphyxia in the observation group were significantly lower than that in the control group (*P* < 0.05), as given in Table 3.

### 3.4. Comparison of Laboratory Indicators of Pregnant Women

Before treatment, there were no significant differences in 24-hour urine protein, random urine protein/creatinine value, serum Hcy, and CRP value of pregnant women in the combination group and routine group; after treatment, the above indexes in the combination group were significantly lower than those in the routine group (*P* < 0.05, Table 4).

### 3.5. Nursing Satisfaction

The nursing satisfaction of the observation group was significantly higher than that of the control group in terms of overall service, environmental comfort, and convenient procedures (*P* < 0.05), as given in Table 5.

## 4. Discussion

Gestational hypertension is one of the major complications of pregnancy and is majorly associated with maternal and fetal death, as well as adverse pregnancy outcomes. The pathogenesis of gestational hypertension is linked to the spasm of the small arteries, which leads to ischemia and hypoxia in the vital organs of the mother, resulting in thick blood, slow blood flow, and ultimately insufficient microcirculation perfusion. Due to the sudden onset and rapid progression of the disease, early detection and early treatment are of huge significance. Clinically, magnesium sulfate mitigates the symptoms of ischemia and hypoxia by exerting central inhibition, antispasmodic, sedative, and vasodilator function. As a commonly used drug for the treatment of hypertension, nifedipine can effectively reduce myocardial oxygen consumption, reduce myocardial contraction, protect the heart muscle, increase coronary blood flow, and decrease blood pressure.

In systematic nursing, medical workers intervene in the patient's diet to ensure that the patient consumes a light diet, with normal dosage of high protein and vitamins and proper intake of calcium, iodine, and other trace elements to reduce the patient's proteinuria, edema, and other pathologies condition. In support of this knowledge, Li et al. [9] pointed out in their study that the systolic blood pressure and diastolic blood pressure in the observation group were lower than those in the control group after treatment, suggesting that nifedipine combined with systematic nursing can effectively mitigate the clinical symptoms of patients and maintain the stability of blood pressure. In line with our hypotheses, we found in the present study that the SDS and SAS scores of the observation group were lower than those of the control group after treatment; the possible explanation may be that on the basis of the drug treatment, the implementation of systematic nursing alleviate the negative emotions of depression and anxiety in patients by communicating with and comforting them, thereby raising their confidence to overcome disease [10]. Similarly, Dai et al. [11] concluded that systematic nursing contributes to eliminate the depression and negative attitude of the patients and boost the enthusiasm and self-confidence of the patients toward treatment by educating health knowledge, implementing psychological nursing, distributing brochures to patients daily, strengthening communication with patients, and answering the questions and doubts of the patients.

In this study, nifedipine and magnesium sulfate were combined for symptomatic treatment of hypertensive patients during pregnancy. The results showed that serum Hcy and CRP values were significantly lower than those in the routine group, which indicates that magnesium sulfate can effectively stabilize blood pressure, reduce peripheral circulatory resistance, and improve brain tissue. Although magnesium sulfate is also commonly used in the treatment of hyperpregnancy, the amount of magnesium ion in the treatment should be noted to achieve the desirable effect. High concentration of magnesium ion adversely impacts the respiratory center and is associated with adverse reactions. On the one hand, by inhibiting the contraction of vascular smooth muscle, it can expand blood vessels, lower blood pressure, and reduce the load on the heart. Nifedipine improves vascular endothelial function, reduces peripheral vascular resistance, and dilates arterioles, with little bearing on postpartum bleeding. On the other hand, it can relax peripheral blood vessels, inhibit the central nervous system, and increase the blood flow of the uterine artery. In addition, the patient's vital signs are regularly monitored in systematic nursing, and urine routine and urine protein are regularly checked, thereby improving pregnancy outcomes and also in keeping with our hypotheses that the incidences of cesarean section, postpartum hemorrhage, premature rupture of membranes, and neonatal asphyxia in the observation group were lower than those in the control group. This would suggest that nifedipine combined with systematic nursing can reduce the occurrence of adverse pregnancy outcomes in patients with gestational hypertension [12]. Also, we found that the complications of uterine atony, neonatal asphyxia, fetal distress, and postpartum hemorrhage in the magnesium sulfate group were lower after treatment, suggesting that systematic nursing + magnesium sulfate in patients with gestational hypertension has a promising clinical efficacy. However, there are still some limitations in this study. First, it was difficult to achieve the standardization and unification of systematic nursing, which needs more special and scientific training. Second, no blind method was adopted in this study, which may bias the research results.

## 5. Conclusion

The implementation of nifedipine plus systematic nursing in patients with gestational hypertension is associated with favorable pregnancy outcome and fewer adverse emotions such as depression and anxiety and superior blood pressure and faster recovery.

## Figures and Tables

**Table 1:** Comparison of blood pressure levels ($\bar{x}$ ± *s*, mmHg).

Groups	Systolic blood pressure		Diastolic blood pressure	
	Before	After	Before	After
Control group (*n* = 60)	158.35 ± 8.67	136.54 ± 10.20	97.85 ± 4.35	85.33 ± 5.01
Observation group (*n* = 60)	157.36 ± 7.58	125.21 ± 7.23	96.53 ± 4.58	78.32 ± 3.54
*t*	0.666	7.020	1.619	8.851
*P*	0.507	<0.001	0.108	<0.001

**Table 2:** Comparison of negative emotion scores ($\bar{x}$ ± *s*).

Groups	SDS		SAS	
	Before	After	Before	After
Control group (*n* = 60)	57.25 ± 5.23	52.31 ± 5.24	52.36 ± 5.36	47.63 ± 5.31
Observation group (*n* = 60)	58.12 ± 5.13	41.23 ± 4.36	52.45 ± 5.61	41.33 ± 5.34
*t*	0.920	12.590	0.090	6.480
*P*	0.360	<0.001	0.929	<0.001

**Table 3:** Comparison of pregnancy outcomes (cases (%)).

Groups	Cesarean section	Postpartum hemorrhage	Premature rupture of membranes	Neonatal asphyxia
Control group (*n* = 60)	35 (58.33)	20 (33.33)	18 (30.00)	15 (25.00)
Observation group (*n* = 60)	15 (25.00)	10 (16.67)	5 (8.33)	3 (5.00)
*χ* ^2^	13.714	4.444	9.090	9.412
*P*	<0.001	0.018	0.001	0.001

**Table 4:** Comparison of laboratory indicators pre and posttreatment ($\bar{x}$ ± *s*).

Groups		24 h urine protein quantification (g/24 h)	Random urine protein/creatinine value (mg/mmol)	Hcy (*μ*mol/L)	CRP (mg/L)
Control group (*n* = 60)	Before	5.05 ± 1.02	540.96 ± 188.0	20.95 ± 2.54	6.41 ± 1.34
	After	1.78 ± 0.84^*∗*^	148.8 ± 49.8^*∗*^	14.02 ± 1.79^*∗*^	2.3 ± 1.13^*∗*^
Observation group (*n* = 60)	Before	5.21 ± 1.40	574.3 ± 1679	21.25 ± 2.71	6.63 ± 2.05
	After	1.22 ± 0.86^*∗*^^∆^	109.4 ± 53.2^*∗*^^∆^	12.16 ± 1.53^*∗*^^∆^	194 ± 0.75^*∗*^^∆^

Compared with before treatment, ^*∗*^*P* < 0.05; compared with the control group, ^Δ^*P* < 0.05.

**Table 5:** Comparison of nursing satisfaction (cases (%)).

Groups	Overall service	Comfortable operation environment	Health education	Convenient procedure	Psychological nursing
Control group (*n* = 60)	54 (90.00)	51 (85.00)	59 (98.33)	54 (90.00)	55 (91.66)
Observation group (*n* = 60)	44 (73.33)	41 (68.33)	46 (76.66)	45 (75.00)	43 (71.66)
*χ* ^2^	5.566	4.658	12.88	4.675	8.015
*P*	0.018	0.031	<0.001	0.031	0.005

## Data Availability

No data were used to support this study.
